# Transforming Growth Factor-β1 Promotes M1 Alveolar Macrophage Polarization in Acute Lung Injury by Up-Regulating DNMT1 to Mediate the microRNA-124/PELI1/IRF5 Axis

**DOI:** 10.3389/fcimb.2021.693981

**Published:** 2021-08-24

**Authors:** Yongqi Wang, Xiaoqing Wang, Hong Zhang, Biao Han, Yuanmei Ye, Mengjie Zhang, Yingbin Wang, Jianjun Xue, Chun’ai Wang

**Affiliations:** ^1^Department of Anesthesiology, The First Hospital of Lanzhou University, Lanzhou, China; ^2^Department of Thoracic Surgery, The First Hospital of Lanzhou University, Lanzhou, China; ^3^Department of Anesthesiology, Lanzhou University Second Hospital, Lanzhou, China; ^4^Department of Anesthesiology, Gansu Provincial Hospital of TCM, Lanzhou, China

**Keywords:** TGFβ1, DNMT1, microRNA-124, PELI1, IRF5, acute lung injury, M1 alveolar macrophage polarization

## Abstract

**Objective:**

Macrophages function as key orchestrators in the pathogenesis of acute lung injury (ALI). The current study sets out to investigate the molecular mechanism of transforming growth factor-β (TGFβ1) in the regulation of M1 alveolar macrophage polarization in ALI by modulating DNA methyltransferase 1 (DNMT1), along with the microRNA (miR)-124/Pellino 1 (PELI1)/interferon regulatory factor 5 (IRF5) axis.

**Methods:**

First, ALI mouse models were established, and the proportion of M1 and M2 macrophages in mouse lung tissues was detected using flow cytometry. The targeting relationship between miR-124 and PELI1 was verified with the help of a dual luciferase gene reporter assay. Following TGFβ1 knockdown, RT-qPCR and Western blot assay were performed to analyze the expression patterns of TGFβ1, DNMT1, miR-124, and PELI1 and M1/M2 polarization markers in the lung tissues of ALI mice. Immunofluorescence was further employed to detect nuclear translocation of IRF5 in macrophages.

**Results:**

The polarization of M1 macrophages was found to be positively correlated with the severity of lung injury. TGFβ1, DNMT1, PELI1 were highly expressed, while miR-124 was down-regulated in ALI mice, and IRF5 was primarily distributed in the nucleus. TGFβ1 promoted the polarization of M1 alveolar macrophages by up-regulating DNMT1. Furthermore, DNMT1 down-regulated the expression of miR-124, which led to enhancement of M1 alveolar macrophage polarization. Meanwhile, over-expression of miR-124 inhibited the nuclear translocation of IRF5 and suppressed M1 alveolar macrophage polarization. On the other hand, over-expression of PELI1 reversed the above trends.

**Conclusion:**

Collectively, our findings indicated that TGFβ1 can promote the expression of DNMT1, which down-regulates miR-124 to activate PELI1 and nuclear translocation of IRF5, thereby aggravating ALI in mice.

## Introduction

Acute lung injury (ALI) is a highly prevalent pulmonary illness, contributing to substantial mortality and morbidity (Abedi et al., 2020). ALI is characterized by the presence of ventilation/perfusion mismatch, serious hypoxemia, as well as poor pulmonary compliance at different degrees (Liu et al., 2021). ALI can be precipitated by a series of intra- and extrapulmonary injury factors, whereas excessive lung inflammation and alveolar epithelial cell apoptosis also play an important role in ALI pathogenesis (Liu et al., 2020). Current evidence further suggests that alveolar macrophages exert crucial functions in ALI, such that macrophage polarization can determine the severity and outcome of disease (Ye et al., 2020). Unfortunately, there is a dearth of treatment modalities against ALI, comprising of lung-protective ventilation, prone positioning, in addition to supportive interventions (Mokra and Mokry, 2021). Therefore, it is imperative to seek novel targets in regard to macrophage polarization for the treatment of ALI.

Transforming growth factor-β (TGFβ) is recognized as a multifunctional cytokine that possesses the ability to mediate various cellular processes, whereas its dysregulation is associated with several diseases (Bizet et al., 2012). In addition, up-regulation of TGFβ1 was previously documented in lung tissues and bronchoalveolar lavage fluid (BALF) collected from neonatal ALI mice (Cheng et al., 2018). Moreover, increased expressions of TGFβ1 by chronic alcohol ingestion in lung fibroblasts are indicated to augment the risk of fibroproliferative damage in ALI mice (Marts et al., 2017). Furthermore, treatment of TGFβ1 can precipitate an increase in DNA methyltransferase 1 (DNMT1) expression in human trabecular meshwork cells (McDonnell et al., 2016). Inherently, DNMT1 plays vital roles in several processes, such as the maintenance of methylation, gene modulation, as well as chromatin stability (Klein et al., 2011). Down-regulation of DNMT1 can further aid in intervening against lung injury under perinatal nicotine exposure (Gong et al., 2015). Meanwhile, studies have also shown that inactivation of DNMT1 signaling contributes to the up-regulation of microRNA (miR)-124 in human oral squamous cell carcinoma cells (Jin et al., 2017). It is noteworthy that over-expression of miR-124 was previously shown to enhance M2 macrophage polarization, thereby dampening ALI (Gu et al., 2017). Further, in regard to macrophage polarization, Pellino 1 (PELI1) is known to promote M1 macrophage polarization by regulating the ubiquitination of interferon regulatory factor 5 (IRF5) and boosting the nuclear translocation of IRF5 (Kim et al., 2017). Interestingly, a prior study indicated that silencing of IRF5 could reverse lung macrophages from the M1 phenotype to M2 phenotype in severe acute pancreatitis-associated ALI (Sun et al., 2016). In lieu of these findings and data, we hypothesized that TGFβ1 could regulate DNMT1 to affect the development of ALI, with the involvement of the miR-124/PELI1/IRF5 pathway, and performed a series of experiments to validate our hypothesis aiming to uncover novel approaches against ALI.

## Materials and Methods

### Establishment of an ALI Model in Mice and TGFβ1 Gene Knockout Mice

Twenty C57BL/6J mice (aged 10–14 weeks) were purchased from the Experimental Animal Center of Southeast University (Nanjing, Jiangsu, China). The obtained mice were allowed to acclimatize to the laboratory conditions for 3 days before the experiment. The mice were individually housed in polypropylene cages and maintained under standard conditions of a constant temperature of 22 ± 2°C and relative humidity of 50 ± 5%, with a 12-h light/dark cycle. The mice were allowed *ad libitum* access to standard laboratory food and water. Lipopolysaccharides (LPS) (*Escherichia coli* O111: B4) were procured from Charles River Laboratories (Margate, Kent, UK). Among the mice, 10 were regarded as the wild type (WT) control mice without treatment, and 10 mice were used to establish the ALI models. First, the randomly selected mice were intraperitoneally anesthetized with 0.1% pentobarbital sodium (50 mg/kg). Subsequently, the vocal cords were identified and isolated by microscopy and external light source. A small catheter was inserted 1 cm below the vocal cords, and then 50 μl LPS (0.5 mg/ml) was dropped onto the trachea. The mice were then suspended in an upright position for 30 s to ensure uniform distribution of LPS in the trachea. Afterward, the animals were placed in a heated oven until they completely recovered from anesthesia.

TGFβ1-gRNA and Cas9 mRNA transcribed *in vitro* were mixed. The mixture was subsequently injected into the cytoplasm of fertilized eggs of specific pathogen-free (SPF) male mice (aged 10–12 weeks, weighing 24–30 g) by microinjection. Next, the surviving fertilized eggs were transplanted into the pseudopregnant recipient mice until childbirth, with the first-generation offspring (F0) obtained. There were eight TGFβ1 knockout mice (gene knockout mice) and eight TGFβ1 WT mice. Specific operation procedures for the construction of TGFβ1 knockout mice were completed by Cyagen Bioscience Inc. (Suzhou, China). Afterward, reverse transcription-quantitative polymerase chain reaction (RT-qPCR) and Western blot assay were performed to detect the expression patterns of TGFβ1 mRNA and protein in the back skin of WT and TGFβ1 knockout mice.

### Determination of Cytokine and Protein Levels in BALF

At the end of the experiment (22–23 h), mice were anesthetized, and BALF samples were obtained by flushing the lungs (1.0 ml) three times. Next, the BALF samples were centrifuged at 1500 rpm for 5 min at 4°C, refrigerated and stored at −80°C. Subsequently, the levels of inflammatory cytokines interleukin-6 (IL-6), tumor necrosis factor-α (TNF-α), and surfactant associated protein A (SP-A) in BALF were detected using enzyme-linked immunosorbent assay (ELISA) kits according to the manufacturer’s instructions.

### Determination of Lung Wet/Dry (W/D) Weight Ratio

At the end of the experiment (22–23 h), the mice were anesthetized with injections of excessive sodium pentobarbital (0.1%, 90 mg/kg), and the mice were euthanized by bloodletting. Lung tissue edema was then estimated by determining the lung W/D weight ratio. The fresh upper part of the right lung tissues was blotted dry before weighing, dried in an 80°C oven for 48 h, and then weighed again to calculate the lung W/D weight ratio.

### RT-qPCR

Total RNA content was extracted from the tissues using the TRIzol reagent (15596026, Invitrogen, Carlsbad, CA, USA). The obtained RNA was reverse-transcribed into complementary DNA (cDNA) according to the instructions of PrimeScript RT reagent kit (RR047A, Takara, Otsu, Shiga, Japan). The synthesized cDNA was subsequently detected with fast SYBR Green PCR kits (Applied Biosystems, Carlsbad, CA, USA) in an ABI PRISM 7500 RT-PCR system (Applied Biosystems), with three replicates set in each well. In addition, the obtained miRNA was reverse-transcribed using miRcute plus miRNA first-strand cDNA synthesis kits (TIANGEN Biotechnology Co., Ltd, Beijing, China) and quantified with miRcute Plus miRNA qPCR detection kits (Tiangen) using specific primers. Glyceraldehyde-phosphate dehydrogenase (GAPDH) or U6 was regarded as the internal parameters, and the relative expression patterns of TGFβ1, DNMT1, PELI1, IRF5, IL-12A, major histocompatibility complex class II (MHCII), CD163, gravity 1 (ARG1), and miR-124 were analyzed using the 2^−ΔΔCt^ method. The primer design is shown in **Supplementary Tables S1, S2**.

### Western Blot Assay

The cells were collected by trypsin digestion and then lysed with enhanced radioimmunoprecipitation assay (RIPA) lysis buffer containing a protease inhibitor (AR0102, Boster, Wuhan, China). Next, the cells were centrifuged at 12,000*g* at 4°C for 15 min, and the supernatant was transferred to a 1.5-ml Eppendorf tube. A bicinchoninic acid (BCA) protein assay kit (AR1110, Boster) was then used to determine the protein concentration. After the addition of protein loading buffer into the supernatant, 20 μg of protein samples were boiled at 98°C for 5 min and subjected to 10% sodium dodecyl sulfate-polyacrylamide gel electrophoresis. Subsequently, the proteins were transferred onto a polyvinylidene fluoride membrane (Millipore Corp., Billerica, MA, USA), which was sealed with 5% bovine serum albumin (BSA) at room temperature for 2 h to block the non-specific binding. The membranes were then incubated overnight at 4°C with diluted rabbit antibodies against TGFβ1 (ab64715, dilution ratio of 1:1000; Abcam, Cambridge, MA, USA), DNMT1 (ab188453, dilution ratio of 1:1000; Abcam), PILI1 (ab199336, dilution ratio of 1:1000; Abcam), IRF5 (ab181553, dilution ratio of 1:1000; Abcam), CD163 (ab182422, dilution ratio of 1:1000; Abcam), ARG1 (ab243892, dilution ratio of 1:1000; Abcam), GAPDH (ab8245; dilution ratio of 1:1000; Abcam), MHCII (86628; dilution ratio of 1:1000; Cell Signaling Technologies, Beverly, MA, USA). Afterward, the diluted horseradish peroxidase (HRP)-labeled secondary antibody goat anti-rabbit (ab6721; dilution ratio of 1:2000; Abcam) or goat anti-mouse (ab6789; 1:2000; Abcam) was incubated with the membranes at room temperature for 1 h. The membranes were developed by enhanced chemiluminescence working liquid (Millipore), and the gray value of each band in Western blot images was quantified using the Image J software, with GAPDH serving as the internal parameter.

### Cell Culture

Human alveolar macrophages were procured from KALANG Biotechnology (#KLH1044, Shanghai, China) and cultured in a humidified incubator (Thermo Fisher Scientific, Rockford, IL, USA) with 5% CO_2_ at 37°C using Rosewell Park Memorial Institute-1640 (RPMI-1640) medium containing 10% fetal bovine serum (FBS; Gibco, Grand Island, NY, USA), 0.37% NaHCO_3_, 100 U/ml streptomycin and 100 U/ml penicillin (Gibco). Meanwhile, mouse alveolar macrophages MH-S purchased from Procell Life Science & Technology Co,. Ltd. (Wuhan, Hubei, China) were cultured in another incubator (Thermo Fisher Scientific) with 5% CO_2_ at 37°C using Ham’s F12K medium (Gibco) containing 15% FBS (Gibco), 100 U/ml streptomycin, and 100 U/ml penicillin. Subsequently, the KLH1044 cells were diluted into a 1 × 10^6^ cells/ml cell suspension, seeded in a 35-mm dish, and cultured in serum-free RPMI-1640 medium containing 100 ng/ml phorbol ester (PMA) and 0.3% BSA for 72 h to induce differentiation. Morphological observation was carried out under a light microscope, and the cells identified to have differentiated into macrophages were selected for subsequent experimentation.

### Cell Transfection

The cells in the logarithmic phase of growth were detached with trypsin and seeded in a six-well plate, at a density of 1 × 10^5^ cells per well. After 24 h of conventional culture, the cells were transfected with 250 μl of Lipo3000 transfection reagent (Invitrogen) at room temperature for 0 to 15 min, and the solution was changed after 16 h. The RNA content was extracted after 48 h, followed by protein extraction after 72 h. The details of experimental grouping were described in the *Results*. mimic-negative control (NC), miR-124 mimic, inhibitor NC, miR-124 inhibitor, sh-NC, sh-TGFβ1, oe-NC, oe-TGFβ1, sh-DNMT1, and oe-DNMT1 were all purchased from Ribobio (Guangzhou, China).

### Hematoxylin and Eosin (HE) Staining

Lung tissues were collected, rinsed with normal saline, drained with filter paper, and sliced into about 1.5-cm pieces. Next, the tissues were fixed with 4% paraformaldehyde, dehydrated, cleared, paraffin-embedded, and sectioned using a slicing machine. Subsequently, the tissue sections were dewaxed, soaked in gradient alcohol, dehydrated, cleared, and sealed with neutral gum. Under a microscope, the nucleus was observed to exhibit blue coloration, and the cytoplasm exhibited pink or red coloration. The staining process was performed according to the instructions of HE staining kits (C0105, Shanghai Beyotime Biotechnology Co. Ltd., Shanghai, China).

### Terminal Deoxynucleotidyl Transferase-Mediated dUTP-Biotin Nick End Labeling (TUNEL) Staining

Apoptosis was detected in the various groups using TUNEL kits (Millipore). First, the lung tissues were rinsed with phosphate-buffered saline (PBS), fixed with 1% paraformaldehyde, and sliced into 4-μm sections. The sections were then stained with fluorescein isothiocyanate (FITC) (green) and 4′,6-diamidino-2-phenylindole (DAPI) (blue) for 10 min. The blue color indicated the nucleus, and the green color indicated the apoptotic cells. Later, apoptosis was observed under a fluorescence microscope (Olympus IX73, Olympus, Tokyo, Japan).

### Flow Cytometry

The distribution of CD86 and CD206 was detected using flow cytometry to determine the ratio of M1/M2 macrophages. Lung single-cell suspension was obtained using a 100-μm filter (Corning Glass Works, Corning, NY, USA) treated with ACK buffer (Thermo Fisher Scientific). Anti-F4/80-APC, anti-CD86-FITC, anti-CD206-PE-Cy5 (eBioscience, San Diego, CA, USA) and negative control immunoglobulin G (IgG) were used for 30 min of staining. The cells were gated on F4/80- and CD86-positive expression, which were identified as the M1 macrophages. In addition, the cells were gated on F4/80- and CD206-positive expression, which were identified as the M2 macrophages. Unstained and fluorescein-conjugated isotypic cells served as the controls. A FACS Calibur (Becton, Dickinson and Company, Franklin Lakes, NJ, USA) flow cytometer was employed for detection, and the data were quantified using the FlowJo software.

### Methylation-Specific PCR (MSP)

Genomic DNA content was extracted from lung tissues and macrophages using QIAamp DNA Mini kits (Qiagen Company, Hilden, Germany), which was transformed into bisulfite with the help of epitect bisulfite kits (Qiagen). The methylation (M) primer sequences were designed as follows: has-miR-124-MF (5′-GTATTTGGGGGTTTATTTTTTGTC-3′), has-miR-124-MR (5′-GAAACCGACTCGAACTTACGTA-3′), mmu-miR-124-MF (5′-ATATAAAGAAGGAGGATTTAGTCGG-3′), mmu-miR-124-MR (5′-CCAAAAATCTAACAAAAAAAACGAA-3′), and the unmethylation (U) primer sequences were: has-miR-124-UF (5′-GTATTTGGGGGTTTATTTTTTGTT-3′), has-miR-124-UR (5′-ATCAAAACCAACTCAAACTTACATA-3′), mmu-miR-124-UF (5′-ATATAAAGAAGGAGGATTTAGTTGG-3′), mmu-miR-124-UR (5′-CCAAAAATCTAACAAAAAAAACAAA-3′). The products were analyzed using agarose gel electrophoresis.

### Dual Luciferase Gene Reporter Assay

The cells were seeded in a 96-well plate upon reaching 70% confluence, and then transfected with luciferase reporter gene plasmids and RNA after 16 h, with three duplicates set in each well. The conditions of transfection were as follows: firefly: Renilla: the transfection reagent = 0.1 μg: 0.01 μg: 0.25 μl; 100 nMRNA and DNA were then incubated at room temperature for 20 min. After removing the medium, 25 μl of DNA transfer mixture and 25 μl of RNA transfer mixture were added to each cell sample, respectively. After 6 h of transfection, the old medium was renewed with fresh complete medium. After 48 h of transfection of mimic-NC and mimic-miR-124, 50 × L diluted 1 × PLB was added to each well, followed by shaking at room temperature for 15 min for lysis purpose. Later, 100 × L of LARII was added to each well of the 96-well enzyme plate with white light transmittance, and then the data were measured after 2 s. Subsequently, 100 μl of Stop & Glo Reagent was added to each well, and then the data was measured again after 2 s in conditions void of light.

### Immunofluorescence

Macrophages were fixed with 4% formaldehyde for 15 min, treated with 0.3% Triton-X100 for 10 min, and then blocked with BSA at 37°C for 1 h, followed by overnight incubation with the primary antibody anti-IRF5 (ab181553; Abcam) at 4°C. Subsequently, the macrophages were incubated with Alexa Fluor-coupled secondary antibody Fluor-488 or -594 goat anti-rabbit or anti-mouse against IgG (ZSGB-BIO, Beijing, China) and Hoechst 33342 at 37°C for 1 h. Afterward, images were acquired using a TCSSP8 confocal microscope (Leica Microsystems Inc., Buffalo Grove, IL, USA). The co-location coefficient of the merged images was processed using the Image-Pro Plus 6.0 software.

### Statistical Analysis

Statistical analyses were performed using the SPSS 21.0 statistical software (SPSS, IBM, Armonk, NY, USA). Measurement data from three independent experiments were expressed by mean ± standard deviation. Data between two groups were compared using independent sample *t*-test, and those among multiple groups were compared using one-way analysis of variance (ANOVA), followed by Tukey *post hoc* test. A value of *p* < 0.05 was indicative of statistical significance.

## Results

### The Severity of ALI Was Positively Correlated With the Proportion of M1 Alveolar Macrophage Polarization

First, we established mouse models of ALI, and then performed ELISA, lung W/D ratio, HE staining, and TUNEL staining to detect whether the model was successfully constructed. It was found that compared with WT mice, ALI mice presented with increased contents of IL-6 and TNF-α in the BALF, lung W/D ratio, and TUNEL-positive cells, whereas the content of SP-A was decreased, in addition to significant lung tissue damage, neutrophil infiltration, and exudation of inflammatory substances in the alveoli, indicating that the ALI mouse models were established successfully (**Figures 1A–D**). Meanwhile, the results of flow cytometry illustrated that only a small number of M1 macrophages were present in the BALF of WT mice, whereas a large number of M1 macrophages were observed in the BALF of ALI mice (**Figure 1E**). Altogether, these findings indicated that the proportion of M1 macrophages was positively correlated with the severity of lung injury.

**Figure 1:** The severity of ALI is positively correlated with the proportion of M1 alveolar macrophage polarization. **(A)** The levels of IL-6, TNF-α, and SP-A in ALI and WT mice were detected by ELISA. **(B)** The lung W/D ratio was calculated to evaluate the severity of pulmonary edema in ALI and WT mice. **(C)** HE staining was used to observe the lung tissue injury in ALI and WT mice. **(D)** TUNEL staining was used to detect lung tissue injury in ALI mice and WT mice (25 μm). **(E)** Flow cytometry was used to detect the ratio of M1 macrophages to M2 macrophages in ALI and WT mice. *p < 0.05 *vs.* WT mice. n = 10.

### TGFβ1 Promoted M1 Alveolar Macrophage Polarization by Up-Regulating DNMT1

To investigate the effect of TGFβ1 and DNMT1 on M1 alveolar macrophage polarization, we first detected the expression patterns of TGFβ1 and DNMT1 in the mouse models using RT-qPCR and Western blot assay. The results illustrated that the expression levels of TGFβ1 and DNMT1 were notably elevated in the lung tissue of ALI mice (**Figures 2A–D**). In addition, relative to WT mice, the lung tissue of ALI mice exhibited a marked increase in the expression levels of M1 macrophage polarization markers IL-12A and MHCII, and a decline in those of M2 macrophage polarization markers CD163 and ARG1 (**Figures 2E, F**).

**Figure 2:** TGFβ1 promotes M1 alveolar macrophage polarization by upregulating DNMT1. **(A)** RT-qPCR was used to detect the mRNA expression of TGFβ1 in lung tissues of ALI mice. **(B)** Western blot assay was used to detect the protein expression of TGFβ1 in lung tissues of ALI mice. **(C)** RT-qPCR was used to detect the mRNA expression of DNMT1 in lung tissues of ALI mice. **(D)** Western blot assay was used to detect the protein expression of TGFβ1 in lung tissues of ALI mice. **(E)** The mRNA expression of M1/M2 polarization markers (IL-12A, MHCII, CD163, and ARG1) of macrophages in ALI mice was analyzed by RT-qPCR. **(F)** The protein expression of M1/M2 macrophage polarization markers (IL-12A, MHCII, CD163, and ARG1) in ALI mice was analyzed by Western blot assay. **(G)** The expression of TGFβ1 and DNMT1 after transfection of sh-TGFβ1 and oe-TGFβ1 was detected by RT-qPCR. **(H)** The expression of M1/M2 polarization markers in human alveolar macrophages KLH1044 with different treatment was detected by RT-qPCR. **(I)** The expression of M1/M2 polarization markers in macrophages MH-S with different treatment was detected by RT-qPCR. *p < 0.05 *vs.* WT mice or sh-NC or sh-NC + oe-NC. ^#^ *p* < 0.05 *vs.* oe-NC or sh-TGFβ1 + oe-NC. n = 10; Cell experiments were repeated three times.

In addition, we up-regulated or down-regulated the TGFβ1 expression in human and mouse macrophage lines. The results of RT-qPCR demonstrated that compared with sh-NC, sh-TGFβ1 decreased the expression levels of TGFβ1 and DNMT; relative to oe-NC, oe-TGFβ1 increased the expression levels of TGFβ1 and DNMT1 (**Figure 2G**). To further explore the effect of DNMT1 over-expression on M1/M2 polarization markers on the basis of silencing TGFβ1 in macrophages, we carried out a rescue experiment. Subsequent results of RT-qPCR displayed that versus sh-NC + oe-NC, sh-TGFβ1 + oe-NC led to significantly decreased expression levels of M1 polarization markers IL12 and MHCII, as well as an increase in those of M2 polarization markers CD163 and ARG1. Moreover, relative to sh-NC + oe-NC, sh-NC + oe-DNMT1 brought about a marked increase in the expression levels of M1 polarization markers IL12 and MHCII, accompanied by a decrease in those of M2 polarization markers CD163 and ARG1. Compared with sh-TGFβ1 + oe-NC, sh-TGFβ1 + oe-DNMT1 led to higher expression levels of M1 polarization markers IL12 and MHCII, in addition to lower expression levels of M2 polarization markers CD163 and ARG1 (**Figures 2H, I**). Overall, these findings suggested that TGFβ1 promoted M1 alveolar macrophage polarization by augmenting the expression of DNMT1.

### DNMT1 Inhibited the Expression of miR-124 and Promoted M1 Alveolar Macrophage Polarization

To explore whether DNMT1 participates in M1 alveolar macrophage polarization by regulating the expression of miR-124, we determined the expression patterns of miR-124 in the mouse models using RT-qPCR. The results illustrated that the expression levels of miR-124 were significantly lower in ALI mice (**Figure 3A**). In addition, MSP assay confirmed that the methylation levels of miR-124 were markedly increased in ALI mice (**Figure 3B**).

**Figure 3:** DNMT1 inhibits the expression of miR-124 and promotes M1 alveolar macrophage polarization. **(A)** RT-qPCR was used to detect the expression of miR-124 in lung tissues of ALI mice. **(B)** MSP assay was used to detect the methylation level of miR-124 in lung tissues of ALI mice. **(C)** RT-qPCR was used to detect the expression of miR-124 in human alveolar macrophages KLH1044 and mouse alveolar macrophage MH-S. **(D)** MSP assay was used to detect the methylation level of miR-124 in human alveolar macrophages KLH1044 and mouse alveolar macrophages MH-S. **(E)** The mRNA expression of M1/M2 polarization markers in macrophages with different treatment was detected by RT-qPCR. **(F)** The protein expression of M1/M2 polarization markers in macrophages with different treatment was detected by Western blot assay. *p < 0.05 *vs.* WT mice or sh-NC or sh-NC + inhibitor-NC. ^#^ *p* < 0.05 *vs.* oe-NC or sh-DNMT1 + inhibitor-NC. n = 10; Cell experiments were repeated three times.

Subsequently, we verified the regulatory effect of DNMT1 on miR-124 using RT-qPCR in human alveolar macrophages KLH1044 and mouse alveolar macrophages MH-S. Based on the results, relative to sh-NC, the expression levels of miR-124 were significantly increased in the presence of sh-DNMT1. Compared with oe-NC, the expression levels of miR-124 exhibited a marked decrease in response to oe-DNMT1 (**Figure 3C**). Meanwhile, MSP assay confirmed that versus sh-NC, sh-DNMT1 led to significantly decreased methylation levels of miR-124; compared with oe-NC, oe-DNMT1 brought about a notable increase in the methylation levels of miR-124 (**Figure 3D**). The results of the rescue experiment in human alveolar macrophages KLH1044 and mouse alveolar macrophages MH-S further revealed that compared with sh-NC + inhibitor NC, sh-DNMT1 markedly inhibited the expression levels of M1 polarization markers of macrophages, whereas miR-124 inhibition brought about the opposite trends. Relative to sh-DNMT1 + inhibitor NC, the expression levels of M1 polarization markers were notably increased in response to sh-DNMT1 + miR-124 inhibitor (**Figures 3E, F**). Overall, these findings suggested that DNMT1 promoted M1 alveolar macrophage polarization by down-regulating miR-124.

### miR-124 Reduced M1 Alveolar Macrophage Polarization by Inhibiting the PELI1/IRF5 Axis

To further elucidate the regulatory mechanism of miR-124 in promoting M1 polarization of macrophages, we predicted the downstream target genes of miR-124 using the starBase (http://starbase.sysu.edu.cn/index.php) and mirDIP (http://ophid.utoronto.ca/mirDIP/index.jsp#r) databases. In addition, we searched the expression microarrays GSE81922 and GSE69607 from the GEO database, with |logFC| > 1 and *p* value < 0.01 serving as the screening standard for differential mRNAs. Using the R language “limma” package, 556 up-regulated and 540 down-regulated mRNAs were screened from the M1 polarization macrophage samples in the GSE81922 microarray; 612 up-regulated and 707 down-regulated mRNAs were screened from the M1 polarization macrophage samples in the GSE69607 microarray (**Figures 4A–D**). The intersection of the abovementioned target genes predicted by the databases and the top 200 up-regulated genes selected by the microarrays was obtained. Only five genes, namely, PELI1, OSBPL3, CPD, PFKFB3, and ACSL1, were found to exist in the four data sets (**Figure 4E**). Remarkably, the PELI1 gene (E3 ubiquitinase) was significantly up-regulated in M1 polarization macrophage samples of the GSE81922 microarray data set (**Figure 4G**).

**Figure 4:** miR-124 reduces M1 alveolar macrophage polarization by inhibiting the PELI1/IRF5 axis. **(A)** The expression heatmap for differential mRNAs in M1 and M2 polarization macrophage samples in GSE81922 microarray. The X-axis represents sample number, the Y-axis represents mRNA, and each small square in the figure represents the expression of one mRNA in one sample. **(B)** Volcano map for expression of differential mRNAs in M1 and M2 polarization macrophage samples in the GSE81922 data set. The black part indicates mRNAs without significant difference, the green part indicates significantly down-regulated mRNAs in M1 polarization macrophage samples, and the red part indicates significantly up-regulated mRNAs in M1 polarization macrophage samples. **(C)** The expression heatmap for differential mRNAs in M1 and M2 polarization macrophage samples in GSE69607 microarray. **(D)** The expression heatmap for differential mRNAs in M1 and M2 polarization macrophage samples in GSE69607 microarray. **(E)** Venn map showing the intersection of the target genes predicted by the starBase and mirDIP databases and the top 200 up-regulated genes selected by the GSE81922 and GSE69607 data sets. **(F)** The binding site of PELI1 and miR-124. **(G)** The expression of PELI1 in M1 and M2 polarization macrophage samples in GSE81922 microarray. **(H)** The binding of miR-124 and PELI1 in macrophages as detected by dual luciferase gene reporter assay. **(I)** RT-qPCR analysis of PELI1 expression in lung tissues in ALI mice. **(J)** Western blot assay analysis of PELI1 expression in lung tissues in ALI mice. **(K)** Immunofluorescence detection of IRF5 localization in macrophages of mouse model. **(L)** Immunofluorescence detection of IRF5 localization in human alveolar macrophages KLH1044 and mouse macrophages MH-S. **(M)** Western blot assay of M1/M2 polarization markers (including IL-12A, MHCII, CD163, and ARG1). *p < 0.05 *vs.* WT mice or mimic-NC or mimic-NC + oe-NC. ^#^ *p* < 0.05 *vs.* miR-124 mimic + oe-NC. n = 10; Cell experiments were repeated three times.

In addition, the results of dual luciferase gene reporter assay illustrated that miR-124 inhibited the PELI1 expression by binding to the PELI1 3′-UTR (**Figures 4F, H**, and **Supplementary Figure 1**). Subsequently, we detected the expression patterns of PELI1 and the localization of IRF5 in the lung tissues of the mouse models. It was found that PELI1 was highly expressed in the ALI mice compared with those in the control mice, and that IRF5 was primarily distributed in the nucleus (**Figures 4I–K**). A rescue experiment in macrophages was then carried out to analyze the regulatory effect of miR-124 on PELI1/IRF5, which demonstrated that over-expression of miR-124 notably inhibited the nuclear translocation of IRF5 and repressed M1 macrophage polarization, whereas PELI1 over-expression brought about the opposite trends. Meanwhile, over-expression of both miR-124 and PELI1 could reverse the effects of miR-124 (**Figures 4L, M**). Collectively, these findings indicated that miR-124 could suppress M1 macrophage polarization *via* inhibition of the PELI1/IRF5 axis.

### TGFβ1 Up-Regulated DNMT1 and Promoted M1 Alveolar Macrophage Polarization Through Mediation of the miR-124/PELI1/IRF5 Pathway

To further verify that TGFβ1 promotes M1 alveolar macrophage polarization by regulating the miR-124/PELI1/IRF5 pathway mediated by DNMT1 *in vivo*, we constructed TGFβ1 gene knockout mice and established mouse models of ALI on this basis. Next, we verified the effect of TGFβ1 gene knockout in the mice, the results of which revealed that TGFβ1 was not expressed in the TGFβ1 knockout mice (**Figure 5A**). Subsequently, the expression patterns of related factors were detected in TGFβ1 knockout mice and WT mice. It was found that compared with WT mice, TGFβ1 knockout mice presented with inhibited expression levels of DNMT1, promoted miR-124 expression levels, and reduced expression levels of PELI1 and nuclear translocation of IRF5 (**Figures 5B, C**). Meanwhile, TGFβ1 knockout mice exhibited lower levels of IL-6 and TNF-α in the BALF and lung W/D ratio, fewer TUNEL-positive cells, higher SP-A levels, attenuated lung tissue damage, reduced neutrophil infiltration, and diminished inflammatory substance exudation in the alveoli relative to WT mice (**Figures 5D–G, I**). Furthermore, the results of flow cytometry illustrated higher number of macrophages of M1 phenotype in the BALF of WT mice than those in the TGFβ1 knockout mice (**Figure 5H**). In conclusion, these findings indicated that TGFβ1 promoted M1 alveolar macrophage polarization by promoting DNMT1 to regulate the miR-124/PELI1/IRF5 pathway.

**Figure 5:** TGFβ1 up-regulates DNMT1 and promotes M1 alveolar macrophage polarization through mediation of the miR-124/PELI1/IRF5 pathway. **(A)** RT-qPCR and Western blot assay were used to detect the expression of TGFβ1 in the lung tissue of WT and TGFβ1 knockout mice. **(B)** The expression of DNMT1, miR-124 and PELI1 in the lung tissue of WT and TGFβ1 knockout mice was detected by RT-qPCR and Western blot assay. **(C)** Nuclear translocation of IRF5 in macrophages was detected by immunofluorescence. **(D)** IL-6, TNF-α, and SP-A levels in the BALF of WT and TGFβ1 knockout mice measured by ELISA. **(E)** Lung W/D ratio measurement in the WT and TGFβ1 knockout mice. **(F)** Lung tissue damage was detected by HE staining (20 μm). **(G)** TUNEL-positive cells in the WT and TGFβ1 knockout mice. **(H)** The proportion of M1 and M2 macrophages detected by flow cytometry in the WT and TGFβ1 knockout mice. **(I)** The expression of M1 and M2 macrophages detected by RT-qPCR. *p < 0.05 *vs.* WT mice. n = 8.

## Discussion

ALI is a continuum of lung changes caused by a variety of lung injuries, which frequently result in significant high morbidity and mortality (Butt et al., 2016). The current study performed a series of *in vivo* and *in vitro* assays to explore the role of TGFβ1 in the progression of ALI, and the obtained findings revealed that TGFβ1 up-regulated DNMT1 to promote M1 alveolar macrophage polarization in ALI *via* the mediation of the miR-124/PELI1/IRF5 pathway.

Initial findings in our study illustrated that the proportion of M1 alveolar macrophage polarization was positively associated with ALI development and that TGFβ1 could promote M1 alveolar macrophage polarization by up-regulating the expression of DNMT1. ALI is characterized as a severe heterogenous pulmonary disorder, with only a handful of therapies (Mokra et al., 2019). Interestingly, promotion of M2 macrophage polarization and diminishing M1 macrophage polarization were previously indicated to aid the attenuation of ALI (Tong et al., 2021). Meanwhile, TGFβ1 is known to trigger mitochondrial dysfunction in alveolar macrophages *via* suppression of the type I IFN response (Grunwell et al., 2018). Similarly, a prior study illustrated that down-regulation of TGFβ1 by N-acetylcysteine conferred protection against cardiopulmonary bypass-induced ALI (Qu et al., 2013). On the contrary, activation of TGFβ1 is known to induce fibrosis after bleomycin-induced ALI, contributing to worse outcomes (Sueblinvong et al., 2014). The hard work done by our peers has further shed light on the interaction between TGFβ1 and DNMT1 in cells, such that TGFβ1 is known to induce the chromatin recruitment of DNMT1 in human hepatic stellate cells (Barcena-Varela et al., 2021). Moreover, TGFβ1 possesses the ability to augment the DNMT1 expression in human trabecular meshwork cells (McDonnell et al., 2016).

In addition, further experimentation in our study demonstrated that DNMT1 inhibited the expression of miR-124, and thus enhanced M1 alveolar macrophage polarization. A number of studies have elaborated the importance of DNMT1 and miR-124 in different lung diseases. For instance, DNMT inhibitor 5-Aza 2-deoxycytidine was previously shown to diminish inflammation while simultaneously augmenting the M2 macrophage phenotype in ALI (Thangavel et al., 2015). Moreover, up-regulated expressions of DNMT1 have been documented in the lung of animals with LPS-induced rhabdomyolysis (Shih et al., 2016). Meanwhile, up-regulation of miR-124 by forsythoside A is also known to regulate macrophage infiltration in lungs to protect against ALI (Lu et al., 2020). What is more, a prior study indicated activation of miR-124-3p because the blockade of SNHG14 could antagonize LPS-induced ALI (Zhu et al., 2021). Intriguingly, a previous study unveiled that miR-124 contributed to amelioration of the lung injury in a mouse model of septic shock (Pan et al., 2019). It is also noteworthy that DNMT1 and miR-124 can interact with each other, such that repression of DNMT1 by amentoflavone contributed to the up-regulation of miR-124-3p in glioma cells (Wang et al., 2018). Furthermore, blockade of DNMT1 because of icaritin treatment was previously indicated to increase miR-124 levels in human oral squamous cell carcinoma cells (Jin et al., 2017).

Moreover, mechanistic experimentation in our study revealed that down-regulation of miR-124 activated the PELI1/IRF5 axis, thereby regulating M1 alveolar macrophage polarization. As previously reported, increased expressions of PELI1 are a common occurrence in patients with frequent exacerbations of asthma or/and chronic obstructive pulmonary disease (Baines et al., 2017). In addition, up-regulated levels of PELI1 in response to LPS and NTHi were previously documented in monocyte-derived macrophages, such that down-regulated PELI1 enhanced immune responses in the airway while promoting bacterial clearance in patients with chronic obstructive pulmonary disease (Hughes et al., 2019). Strikingly, inhibition of IRF5 was previously suggested to suppress chronic macrophage-induced inflammation and alleviate lung injury (Weiss et al., 2015). IRF5, as a marker of proinflammatory macrophages, can be down-regulated by SB203580, whereas its resultant inhibition is known to aid in protecting against inflammation and lung injury induced by LPS (Li et al., 2020). Nevertheless, the regulatory relationship between miR-124 and PELI1/IRF5 requires much exploration. However, existing evidence suggests that PELI1 can interact with IRF5 in the cytoplasm, leading to increased nuclear translocation of IRF5 through K63-linked ubiquitination in M1 macrophages, thereby regulating glucose intolerance in obesity (Kim et al., 2017).

## Conclusion

Altogether, the current study demonstrated that TGFβ1 can up-regulate DNMT1, resulting in down-regulation of miR-124 to augment the expression of PELI1 and nuclear translocation of IRF5, which consequently aggravates ALI in mice (**Figure 6**). Our findings provide a new theoretical basis for understanding the function of TGFβ1 in the progression of ALI. However, further exploration is still warranted to validate the clinical feasibility of our findings and improve diagnostic and therapeutic modalities for ALI.

**Figure 6:** The molecular mechanism plot. TGFβ1 induces the expression of DNMT1, which down-regulates miR-124 to promote the expression of PELI1 and nuclear translocation of IRF5, thereby eventually aggravating ALI in mice.

## Data Availability Statement

The original contributions presented in the study are included in the article/**Supplementary Material**. Further inquiries can be directed to the corresponding author.

## Ethics Statement

The current study was approved by the ethics committee of The First Hospital of Lanzhou University. Animal experimentation protocols were evaluated and approved by the ethics committee of The First Hospital of Lanzhou University. Extensive efforts were made to minimize the number and suffering of the experimental animals.

## Author Contributions

YQW and XW conceived and designed research. HZ performed experiments. BH and YY interpreted results of experiments. MZ analyzed data. YBW prepared figures. JX drafted paper. CW edited and revised manuscript. All authors contributed to the article and approved the submitted version.

## Funding

This work is supported by Natural Science Foundation of Gansu Provincial Science and Technology Department (17JR5RA264).

## Conflict of Interest

The authors declare that the research was conducted in the absence of any commercial or financial relationships that could be construed as a potential conflict of interest.

## Publisher’s Note

All claims expressed in this article are solely those of the authors and do not necessarily represent those of their affiliated organizations, or those of the publisher, the editors and the reviewers. Any product that may be evaluated in this article, or claim that may be made by its manufacturer, is not guaranteed or endorsed by the publisher.

## Supplementary Material

Supplementary Table 1 The expression of miR-124 and PELI1 in human and mouse alveolar macrophages.
